The article "Amodiaquine-Artesunate versus Artemether-Lumefantrine against Uncomplicated Malaria in Children Less Than 14 Years in Ngaoundere, North Cameroon: Efficacy, Safety, and Baseline Drug Resistant Mutations in pfcrt, pfmdr1, and pfdhfr Genes" was retracted in 2019. Reasons: errors in the methods; no approval from the institution; no approval from a third party.

# Amodiaquine-Artesunate versus Artemether-Lumefantrine against Uncomplicated Malaria in Children Less Than 14 Years in Ngaoundere, North Cameroon: Efficacy, Safety, and Baseline Drug Resistant Mutations in *pfcrt*, *pfmdr1*, and *pfdhfr* Genes

**DOI:** 10.1155/2013/234683

**Published:** 2013-12-15

**Authors:** Innocent M. Ali, Palmer M. Netongo, Barbara Atogho-Tiedeu, Eric-Olivier Ngongang, Anthony Ajua, Eric A. Achidi, Wilfred F. Mbacham

**Affiliations:** ^1^Laboratory for Public Health Research Biotechnologies, University of Yaounde, BP 8094, Yaounde, Centre Region, Cameroon; ^2^Department of Biochemistry, University of Dschang, BP 67, Dschang, West Region, Cameroon; ^3^Universite des Montagnes, BP 208, Bangante, West Region, Cameroon; ^4^Faculty of Science, University of Buea, BP 63, Buea, South West Region, Cameroon

## Abstract

*Background*. In Cameroon, both Artesunate-amodiaquine (AS/AQ) and artemether-lumefantrine (AL) are used as first-line treatment against uncomplicated malaria in line with the WHO recommendations. We compared the efficacy and safety of both therapeutic combinations and determined the prevalence of drug resistance conferring mutations in three parasite genes. *Methods*. One hundred and fifty acute malaria patients between six months and 14 years of age were randomized to receive standard doses of either AS/AQ (73) or AL (77) and followedup for 28 days. Outcome of treatment was according to the standard WHO classification. DNA samples from pretreatment parasite isolates were used to determine the prevalence of resistant mutations in the *pfcrt*, *pfmdr1*, and *dhfr* genes. *Results*. Both drug combinations induced rapid clearance of parasites and malaria symptoms. PCR-corrected cure rates were 100% and 96.4% for AL. The combinations were well tolerated. Major haplotypes included CVIET (71%), CVMNT (25%) for the *pfcrt*; SND (100%) for the *pfmdr1*; IRN (79, 8%), NCS (8.8%), and mixed haplotype (11, 8%) for the *dhfr*. *Conclusion*. Both AS/AQ and AL were highly effective and well tolerated for the treatment of uncomplicated falciparum malaria in Ngaoundere, Cameroon. High prevalence of mutant *pfcrt* alleles confirms earlier observations. Long-term monitoring of safety and efficacy and molecular markers is highly solicited.

## 1. Introduction

Malaria remains one of the most serious health problems worldwide and a leading cause of childhood morbidity and mortality in Africa [1]. Early diagnosis and prompt effective treatment remains the cornerstone for the reduction of malaria-related morbidity and mortality [2]. The control of malaria has been challenged by increasing resistance of *Plasmodium falciparum* to antimalarial drugs, particularly chloroquine (CQ) and sulfadoxine-pyrimethamine (SP), leading to sweeping changes in antimalarial treatment recommendations [3]. However, the decision to change antimalarial treatment guidelines is complex. This is limited by the ready availability of alternatives with proven clinical efficacy, procurement and supply costs, and likely durability of the new policy. The latter is largely determined by the rate at which resistance to the first-line drugs develops, itself a function of the mechanisms of resistance to the antimalarial.

The article "Amodiaquine-Artesunate versus Artemether-Lumefantrine against Uncomplicated Malaria in Children Less Than 14 Years in Ngaoundere, North Cameroon: Efficacy, Safety, and Baseline Drug Resistant Mutations in pfcrt, pfmdr1, and pfdhfr Genes" was retracted in 2019. Reasons: errors in the methods; no approval from the institution; no approval from a third party.

Across Africa, *P. falciparum* resistance to the inexpensive and widely used drugs has reached very high levels, and noticeably hampered malaria control efforts in the region [3–5]. As a consequence, the use of combination therapy against malaria has been widely advocated and now implemented in a majority of endemic African countries [6]. Combination regimens, including a number of artemisinin-based combination therapies (ACTs), have replaced monotherapies for treatment of uncomplicated malaria. They are preferred because artemisinin compounds have rapid fever and parasite clearance effects and also reduce gametocyte rate with the potential to reduce transmission and are generally well tolerated [7, 8].

Since April 2001, WHO recommended the use of ACTs in countries where *P. falciparum *malaria is resistant to CQ, SP, and amodiaquine (AQ). Two of the four ACTs recommended by WHO [9], artemether-lumefantrine and artesunate + amodiaquine, have recently been adopted as first-line therapy by many countries in sub-Saharan Africa. At present, 60 countries have adopted ACTs as recommended by the WHO, and 33 countries including Cameroon are deploying ACTs to the peripheral health services [10].

In Cameroon, an interim policy was adopted involving the use of AQ as the first line drug for uncomplicated malaria [11]. As a consequence CQ was abandoned and withdrawn from the official drug outlets in Cameroon [12]. Due to decreased sensitivity of *P. falciparum *to AQ and SP in the country, the Ministry of Health of Cameroon decided to revise its treatment policy as recommended by WHO and replaced AQ with artemisinin-based combination with resources from the Global Fund. The current treatment protocol for uncomplicated *falciparum* malaria in Cameroon is artesunate plus amodiaquine, and artemether-lumefantrine as first-line treatment for uncomplicated falciparum malaria. However, which regimens offer optimal therapies for malaria in Cameroon at that time was unclear.

As of 2007, few studies on the efficacy on AS/AQ had been conducted in the country. In 2008, Ndiaye et al. [13] in a pilot multicentre study confirmed the efficacy and good tolerability of artesunate plus amodiaquine. Although this multisite 14 days protocol study reported high efficacy to both combinations, the efficacy evaluations were done within a limited follow-up time (14 days) and so had some potential to underestimate treatment effects. More importantly, it did not show whether the small proportion of treatment failures observed was due to a recrudescence of existing parasites or acquisition of a new infection; except for the latter which reported a 99.4% PCR-corrected efficacy of artesunate plus amodiaquine.

The article "Amodiaquine-Artesunate versus Artemether-Lumefantrine against Uncomplicated Malaria in Children Less Than 14 Years in Ngaoundere, North Cameroon: Efficacy, Safety, and Baseline Drug Resistant Mutations in pfcrt, pfmdr1, and pfdhfr Genes" was retracted in 2019. Reasons: errors in the methods; no approval from the institution; no approval from a third party.

Considering the urgent need for reliable data on the efficacy and safety of ACTs at that time, the efficacy, safety, and tolerability of two presumably highly efficacious ACTs (artesunate plus amodiaquine and artemether plus lumefantrine) for the treatment of malaria in Cameroon were evaluated within the 28 days efficacy protocol based on the WHO 2003 guidelines for evaluation of drug efficacy [14]. The primary objective of the study was therefore to evaluate the clinical and efficacy, safety and tolerability of the first-line artemisinin-based drug combinations in the treatment of uncomplicated malaria due to *P. falciparum *in Ngaoundere, Cameroon. Secondly, we set out to determine the baseline prevalence of mutations in the *pfcrt, pfmdr1,* and* dhfr* genes in parasites circulating in the study area for subsequent drug efficacy and resistance surveillance countrywide.

## 2. Materials and Methods

### 2.1. Study Site

This study was conducted in 2007 between September and December at the Ngaoundere Protestant Hospital, which is one of two general hospitals in Ngaoundere. Ngaoundere is the chief town of Adamawa Province of Cameroon located in the mid-northern half of the country and generally characterized by savanno-sahelian geography, tropical climate with 2 distinct seasons, and seasonal malarial transmission periods. The main vector is *Anopheles funestus *and the number of infective bites associated with *Plasmodium falciparum *is estimated at <10 per person per year. Crude malaria prevalence rate in children less than five years was estimated at about 12% according to the 2006 National Malaria Control Programme report [13]. In 2008, malaria morbidity was estimated at 35% in the Adamaoua region whose capital in Ngaoundere. Close to 10% of all uncomplicated malaria cases progressed to severe malaria in this region (http://www.casecameroon.org/case/images/documentation/epidemiology/THE%20CAMEROON%20MALARIA%20REPORT.pdf). Ngaoundere is considered as one of the surveillance sites for antimalarial drug efficacy in Cameroon.

### 2.2. Study Design

This study was an open label, randomized controlled trial comparing the efficacy, safety, and tolerability of artesunate plus amodiaquine (coblister) and artemether-lumefantrine (FDC) in a population of children 6 months to 14 years of age following the standard WHO 2003 efficacy assessment protocol [14].

The article "Amodiaquine-Artesunate versus Artemether-Lumefantrine against Uncomplicated Malaria in Children Less Than 14 Years in Ngaoundere, North Cameroon: Efficacy, Safety, and Baseline Drug Resistant Mutations in pfcrt, pfmdr1, and pfdhfr Genes" was retracted in 2019. Reasons: errors in the methods; no approval from the institution; no approval from a third party.

### 2.3. Sample Size Determination

To determine the sample size required to demonstrate no difference in proportion of adequate clinical responses between the AS/AQ group and the AL group (intergroup difference <10%) in the total population with a type I error of 5% and a power of 80% to be able to detect such a difference. The minimal sample size determined also to obtain results that were meaningful and cost effective to the ministry of public health was 60 per group. With a loss to follow-up rate estimated at 20%, we arrived at a total of 150 patients; 75 per treatment arm.

### 2.4. Patients

The study included sick children who were six months to 14 years old if they presented with an axillary temperature of ≥37.5°C or a history of fever in the past 24 hours and monoinfection with *P. falciparum* count of 1,000–200,000 parasites/*μ*L. Children were excluded if they presented with the following: severe *falciparum *malaria, documented intake of AS/AQ or AL, or another antimalarial drug two weeks preceding enrolment (including cotrimoxazole), other causes of fever, evidence of underlying chronic diseases (cardiac, renal, hepatic, and malnutrition), history of allergy to study drugs or known allergy to other antimalarial drugs, residence out of the study area, patient's parent/guardian unwillingness to provide written informed consent, and inability to take oral medication. Other exclusion criteria included development of concomitant disease which would interfere with the classification of treatment outcome. Patients were withdrawn from the study if any of the following occurred: (1) use of antimalarial drugs outside of the study protocol; (2) concomitant febrile illness; (3) withdrawal of consent; (4) protocol violation; and (5) loss to followup. Patients that did not return on schedule for followup were visited at home on the same day.

### 2.5. Randomisation and Treatment

After inclusion, patients were weighed then allocated to either of the two treatment arms. Randomisation was done in blocks of 10 according to a preestablished list with random numbers and sequences generated electronically. Each block was a sealed envelope containing serially arranged codes according to the sequence of randomization by a data manager. Dosages of the study drugs were as follows: (1) 4 mg/kg/day artesunate plus 10 mg/kg/day amodiaquine, for 3 days and (2) artemether-lumefantrine: six doses consisting of two daily doses for 3 days. The dosages were adjusted according to the weight of the patient to the nearest quarter of a tablet.

The article "Amodiaquine-Artesunate versus Artemether-Lumefantrine against Uncomplicated Malaria in Children Less Than 14 Years in Ngaoundere, North Cameroon: Efficacy, Safety, and Baseline Drug Resistant Mutations in pfcrt, pfmdr1, and pfdhfr Genes" was retracted in 2019. Reasons: errors in the methods; no approval from the institution; no approval from a third party.

Treatment allocation was concealed until final enrolment of the patient by the study physician. Drug administration was directly observed by the study nurse or pharmacist for 30 minutes. Children who vomited within 30 minutes received a second dose. If vomiting persisted, the child was excluded from the study. For AL, the morning doses were directly observed over the 3 days of treatment, while the evening doses were given to the patients to be taken at home, and empty sachets returned as evidence of ingestion of the drug. AL was administered with a cup of milk (3% fat). Each parent or guardian of a participant was advised to administer home doses of AL as observed in the hospital and to report to the hospital if the child vomited or refused to take the medication. We also encouraged the parents or guardians to return to the hospital any time they feel concerned about anything.

### 2.6. Clinical and Laboratory Procedures

Patients were scheduled for follow-up examinations on days 1, 2, 3, 7, 14, and 28 and any other time the participant felt unwell during the study period. On each visit, complete physical and clinical examinations as well as biological evaluations were performed. Patients or guardians were asked about drug consumption and visits to the local pharmacy since the last clinic visit. Children who failed treatment were rescued with quinine tablets/or infusion according to the local treatment guidelines.

Giemsa stained thick and thin blood smears were prepared on days 0, 1, 2, 3, 7, 14, 28, and any time there was a health concern or fever. Asexual parasites were counted against 200 leucocytes and the parasite density expressed as per *μ*L of blood, assuming a mean value of 8,000 leucocytes/mm^3^ of blood. At least 100 thick film fields were examined before a slide was considered negative. The parasite speciation was determined on the thin blood film. In addition, venous blood specimen (3–5 mL in EDTA tubes) obtained on days 0 and 14 from the enrolled individuals was used to determine a complete blood counts (haemoglobin [Hb], WBC & RBC counts, and WBC differential count) on a Coulter 890 instrument (Coulter Corp., Miami, FL). Blood collected in dry tubes was used for biochemical analyses (alanine aminotransferase—ALT, total bilirubin, and Creatinine) measured using a Kodak Ektachem DT-60 automatic system (Eastman Kodak Co., Rochester, NY). This was done on samples collected from all patients as part of the safety assessment at baseline and selected days during followup.

Filter-paper blood spots (Whatmann No. 3chromatography filter paper) collected from finger pricks on day 0 and on the day of recurrent fever/parasitaemia were used for molecular genotyping to distinguish recrudescence from new infection for all patients and those failing therapy. Briefly, parasite DNA extracted from filter paper blood spots was analysed for length polymorphisms in the gene encoding merozoite surface protein-1 (*MSP 1*) and merozoite surface protein-2 (*MSP 2*) using nested PCR. First, *MSP 2* genotyping patterns on the day of failure were compared with those before treatment initiation. If all of the *MSP 2* alleles present on the day of failure were present at the time of treatment initiation, genotyping was repeated using *MSP 1*. An outcome was defined as recrudescence if all *MSP 1* and *MSP 2* alleles present at the time of failure were present at the time of treatment initiation and defined as a new infection as previously described [15]. Baseline prevalence of molecular markers of resistance was estimated after PCR-RFLP on extracted DNA samples as previously described [16, 17]. Haplotypes were constructed from combinations of point mutations for each sample. They were classified as resistant, mixed, or sensitive based on whether the haplotype represented combinations of resistance related mutations, mutant and nonmutant forms, or wild type alleles of the gene encoding the drug target in question.

The article "Amodiaquine-Artesunate versus Artemether-Lumefantrine against Uncomplicated Malaria in Children Less Than 14 Years in Ngaoundere, North Cameroon: Efficacy, Safety, and Baseline Drug Resistant Mutations in pfcrt, pfmdr1, and pfdhfr Genes" was retracted in 2019. Reasons: errors in the methods; no approval from the institution; no approval from a third party.

### 2.7. Classification of Treatment Outcomes

The primary efficacy endpoint was day 28 cure rate of both drugs, which was defined as the proportion of patients clearing their asexual parasites without recrudescence within the 28-day trial period. The day-28 cure rate was adjusted on the basis of the PCR genotyping results of paired samples for patients with recurrent parasitaemia between days 4 to 28. Outcome of treatment was defined according to the standard WHO classification as follows: early treatment failure (ETF); late clinical failure (LCF); late parasitological failure (LPF), and adequate clinical and parasitological response (ACPR). Total treatment failure was considered to be sum LCF and LPF and classified based on PCR confirmed recrudescence of recurrent parasitaemia.

Secondary efficacy endpoints included fever clearance, parasite clearance, and day 14 haemoglobin recovery. The primary safety endpoint was the incidence of adverse events in both groups, clinical and biological drug safety and tolerance An adverse event was defined according to ICH guidelines as any untoward sign, symptom, intercurrent illness, or abnormal laboratory value not present on day 0 but which occurred during followup or was present on day 0 and became worse during follow-up resulting in the withdrawal of the participant from the study, hospitalization, or death. All adverse events (AEs) were classified according to the common toxicity criteria, recorded on the Case Report Form (CRF) and treated according to standard medical guidelines. Data on adverse events was evaluated by an independent data safety and monitoring board that oversaw the trial enrolment progress.

The article "Amodiaquine-Artesunate versus Artemether-Lumefantrine against Uncomplicated Malaria in Children Less Than 14 Years in Ngaoundere, North Cameroon: Efficacy, Safety, and Baseline Drug Resistant Mutations in pfcrt, pfmdr1, and pfdhfr Genes" was retracted in 2019. Reasons: errors in the methods; no approval from the institution; no approval from a third party.

### 2.8. Ethical Statement

The local health and institutional authorities approved the research protocol (Cameroonian Ministry of Public Health) and delivered an ethical clearance. Signed informed consent for participation was obtained from parents or guardians for their children, after they were adequately informed of study objectives, detailed procedures including any associated discomfort, and ultimate benefits of the study to the wider community. This information was provided in the local language (Fulfulde), French, or English. Parents or guardians were also informed they were free to withdraw their children from the study at any time without prior notice or consequence on the quality of health care received by their children. The contact address of local institutions (administrative and ethics) authorising the study was provided in case the participants desired independent information on the study.

### 2.9. Data Analysis

Data recorded in each patient's CRFs comprised information on demography, parasite counts, signs and symptoms, laboratory data, concomitant infection/treatment, and adverse events for each scheduled visit. These were double keyed in Excel (Microsoft Corporation, Redmond USA 2003) by two data technicians. Reconciled data were then exported to SPSS version 9.0 for further analysis. Data of the patients excluded or lost to followup were censored at the time of the last recorded visit. Descriptive statistics presented as counts, percentages, means, and standard deviations, as appropriate, were used to compare the demographic characteristics of the study population and their initial clinical and biological characteristics (such as temperature and geometric mean parasitaemia).

Primary efficacy analysis which represented evaluating differences in proportions of treatment outcome was done using the chi-squared test (*χ* ^2^) or Fisher's exact test. The two-tailed Student's *t*-test was used to compare group means with a 95% confidence interval for both secondary efficacy and primary safety analysis. A difference in outcome measure was considered statistically significant when the *P* value was less than the cut off (0.05). Primary efficacy was assessed as per protocol (PP), using the Kaplan Meier survival curve with hazard ratios to compare primary outcome between groups. New infections were censored from the data using this analysis. The study was carried out according to the principles of good clinical and laboratory practices.

The article "Amodiaquine-Artesunate versus Artemether-Lumefantrine against Uncomplicated Malaria in Children Less Than 14 Years in Ngaoundere, North Cameroon: Efficacy, Safety, and Baseline Drug Resistant Mutations in pfcrt, pfmdr1, and pfdhfr Genes" was retracted in 2019. Reasons: errors in the methods; no approval from the institution; no approval from a third party.

## 3. Results

### 3.1. Baseline Characteristics

A total of 150 children were recruited during the 5-months study period. Of these, 73 were randomized to AS/AQ and 77 to artemether-lumefantrine (AL). Of all randomised patients, 137 were seen on day 14 and 125 on day 28. Altogether, 61 (83.6%) completed the study after treatment with AS/AQ and 64 (83.1%) with AL.

No significant differences in sex, age, weight, temperature haemoglobin levels, parasite density, and anaemia status between AS/AQ group and the AL group existed (Table 1). There were 78 (52%) male and 72 (48%) female patients enrolled in this study. Their overall mean (±SD) age, weight, and temperature values were 04.95 (±3.47) years, 16.6 (±7.66) kg, and 37.9 (±1.002)°C. The geometric mean baseline parasitaemia was 4231 parasites/*μ*L of blood. With respect to age 56% of patients were ≤ 5 years of age, and 44% were 6–14 years of age. Using these categories there was no difference between response to the two drugs used and number of subjects in each category (*P* > 0.05).

### 3.2. Primary Outcome: Day 28 Cure Rates for Both Treatments

In both treatment groups, most of the participant completed the 28-day followup and were included in the study analysis. Losses to follow-up were 13 (5 AS/AQ, 8 AL) by day 14, and a further 12 (7 AS/AQ, 5 AL) by day 28. The results of the treatment efficacy are presented by treatment group and day of followup, unadjusted and adjusted by genotyping (Table 2). At day 14, cure rates with AL was better compared with that for AS/AQ. Cure rates decreased during followup in the two treatment groups. However, at day 28, the A/L group was highly effective to treat *P. falciparum *infections and prevent parasite reemergence than participants of the AS/AQ group. Only nine treatment failures were observed: seven (11.5%) in the AS/AQ group and two (03.1%) in the AL group. Most of the therapeutic failures were classified as LPF (AS/AQ group) and on or before day 7 (AL group). All failure samples were genotyped and classified as either reinfection or recrudescence. After PCR correction and exclusion of reinfections, AS/AQ resulted in 03.6% (02/56) confirmed failures and no true failure with AL. Excluding seven protocol violations, 56 (AS/AQ) and 62 (AL) were included in the Kaplan Meier analyses.

Figure 1 shows the Kaplan-Meier curve of cumulative treatment success over the 28-day follow-up period, adjusted by genotyping.

The hazard rate for the first three days of treatment was 2/61 (0.03) for participants in the AS/AQ group and 0/69 (0) for the AL group. Beyond this point, no treatment failure occurred when the outcome measures were corrected by PCR in the per protocol analysis.

The article "Amodiaquine-Artesunate versus Artemether-Lumefantrine against Uncomplicated Malaria in Children Less Than 14 Years in Ngaoundere, North Cameroon: Efficacy, Safety, and Baseline Drug Resistant Mutations in pfcrt, pfmdr1, and pfdhfr Genes" was retracted in 2019. Reasons: errors in the methods; no approval from the institution; no approval from a third party.

### 3.3. Secondary Efficacy Outcomes: Fever and Parasite Clearances, Haematological Recovery, and Biological Tolerance

#### 3.3.1. Fever Clearance

Children who received AL were more likely to be febrile (axillary temperature ≥ 37.5°C) on days 1 (15/77) and 28 (02/64) than those treated with AS/AQ (day 1; 12/73 versus 01/61 on day 28). More fever clearance in the AL treatment group did not, however, translate into a clear clinical benefit since there was no consistent difference in the pattern of fever clearance between the 2 treatment groups (*P* > 0.05 at each contact; Figure 2).

#### 3.3.2. Parasite Clearance

The rate of parasite clearance was similar in the two groups during the first 7 days (Figure 3). Although children who received AS/AQ appeared to clear parasites faster as seen on days 2 and 3 compared to children in the AL group, the difference in the number of parasitaemic children in both groups was not significant (*P* > 0.05). Subsequently, after day 7, parasite clearance was clearly superior in the AL treatment group, with no cases associated with a positive blood smear result by days 14 and 28 compared with 1.8% and 5.3% in the AS/AQ group (*P* < 0.001, Figure 3).

#### 3.3.3. Clinical and Biological Tolerance to Treatment

At enrolment, patients in both treatment groups showed symptoms common to malaria such as headache, asthenia, fatigue, fever, dizziness, nausea, myalgia, and anorexia. Other less commonly observed symptoms/signs included rigors, arthralgia, vomiting, sleep disorders, and abdominal pain. As anticipated, the malaria symptoms disappeared rapidly within 2–5 days in most of the patients in both treatment groups.

Adherence to treatment was generally good. Artemether-lumefantrine and AS/AQ were well tolerated. Complete safety records were available for 137 (AS/AQ; 68 and AL; 69) patients enrolled into this study. No serious AEs were observed or reported during followup and none of the failures developed into complicated malaria. However, abnormalities in laboratory results (leukopenia, neutropenia and anaemia) were common after treatment with AS/AQ (33.8%; 23/68) and AL (30.4; 21/69) but similar in the two arms (Table 3).

No severe alterations in renal or hepatic function were observed with any of the drug combinations under study, although increase in bilirubin, creatinine and ALT was observed. The observed day 14 increase in transaminase did not exceed the critical threshold and so was of limited clinical significance. Only two patients, one treated with AS/AQ and the other in the AL group presented with a slight transient increase in alanine transaminase and creatinine, levels, respectively. These changes were not accompanied by clinical signs and therefore had no definite therapeutic implications.

The article "Amodiaquine-Artesunate versus Artemether-Lumefantrine against Uncomplicated Malaria in Children Less Than 14 Years in Ngaoundere, North Cameroon: Efficacy, Safety, and Baseline Drug Resistant Mutations in pfcrt, pfmdr1, and pfdhfr Genes" was retracted in 2019. Reasons: errors in the methods; no approval from the institution; no approval from a third party.

#### 3.3.4. Haematological and Biochemical Changes

At day 14 after treatment, 125 (*n* = 68, AS/AQ; *n* = 69, AL) patients had paired day 0/day 14 haematological and biochemical clinical values (Table 4). In patients treated with AS/AQ, there were no significant changes in mean values between day 0 and day 14 for the haemoglobin (*P* = 0.52), haematocrit (*P* = 0.87), total red blood count (RBC) (*P* = 0.65), and other red cell indices (*P* > 0.05). However, there was a significant decrease of total WBCs from day 0 to day 14 (*P* = 0.04) as well as an increase of platelet count from day 0 to day 14 (*P* = 0.001). The mean ALT decreased slightly during followup but there was no significant decrease from day 0 to day 14 while there was a small but not statistically significant increase in the mean creatinine and bilirubin values between day 0 and day 14 (Table 4).

Similarly, patients treated with AL showed no significant changes in mean values between days 0 and 14 for the haemoglobin (*P* = 0.70), haematocrit (*P* = 0.66), total RBC (*P* = 0.96), and red cell indices (*P* > 0.05). Also, a significant decrease in total WBC (*P* = 0.025) and a significant increase (*P* = 0.002) for platelet count was observed from day 0 to day 14 during followup. Mean ALT and bilirubin were found to decrease slightly during follow-up but there were no significant decreases from day 0 to day 14 while there was a small (0.83) but statistically significant increase in the mean creatinine value between day 0 and day 14 (Table 4).

Taken together, the mean values of routine haematological and biochemical variables were similar in the two study groups and there were no significant differences in the proportions of children with abnormal biochemical test results in the two drug groups.

#### 3.3.5. Prevalence of *pfcrt*, *pfmdr1*, *dhfr*, and *dhps* Haplotypes

Mutations defining haplotypes in the *pfcrt, pfmdr1*, and *pfdhfr* genes were genotyped and baseline prevalence obtained. High level resistant haplotypes in the *pfcrt* included CVIET (71%) and CVMNT (25%) while 4.5% of the isolates contained mixed genotypes. Point mutations in the *pfmdr1* were all of the wild type defining the haplotype SND (100%). The haplotypes in the *dhfr *included the triple mutant IRN observed at high frequency (79.8%) as opposed to the wild type (NCS) observed at very low frequency (8.8%). These results are summarised in Figure 4.

The article "Amodiaquine-Artesunate versus Artemether-Lumefantrine against Uncomplicated Malaria in Children Less Than 14 Years in Ngaoundere, North Cameroon: Efficacy, Safety, and Baseline Drug Resistant Mutations in pfcrt, pfmdr1, and pfdhfr Genes" was retracted in 2019. Reasons: errors in the methods; no approval from the institution; no approval from a third party.

Eleven percent of infections consisted of the mixed haplotype for the *dhfr.* Resistant haplotype SGK was low (25.5%) compared to the sensitive haplotype SAK (55.7%). There were no differences in the proportion of children carrying mutant haplotypes between treatment groups.

## 4. Discussion

### 4.1. Primary Outcome

Artemisinin-based combination therapy (ACT) is being widely promoted as a strategy to counteract increasing resistance of *P. falciparum *to antimalarial drugs [9]. This is because the artemisinin derivatives are highly effective antimalarial compounds against the different stages of *Plasmodium *development [7]. In order to prolong the efficacy of these drugs, it is recommended that they should only be used in combination with another effective drug that has a longer half-life. In this light, AS/AQ and AL were chosen as the recommended treatments for first- and second-line treatments for uncomplicated malaria. The main goal of this *in vivo *ACT efficacy study was to evaluate the clinical efficacy, safety, and tolerability of AS/AQ and AL in Ngaoundere, a savannah region in the north of Cameroon with moderate to high incidence of *P. falciparum *malaria. The results of this study demonstrated that the two artemisinin drug regimens tested had good clinical and parasitological efficacy. Cure rates of the two combinations were high (3-dose AS/AQ (88.5%) and the 6-dose regimen of AL (96.9%)) with a total of seven and 2 cases with recurrent parasitaemia in the AS/AQ and AL treatment groups respectively. Most of these recurrent parasitaemia samples were reclassified as reinfections based on PCR genotyping. Both crude and PCR-corrected ACPRs for AL (96.9% and 100%) were higher than those recorded in the AS/AQ (88.5% and 96.4%) arm. Artemether-lumefantrine appeared to be the better treatment option on the basis of non-PCR corrected responses, based on the lower percentage of recurrent parasitaemia observed. The PCR corrected cure rates indicated the true efficacy is comparable between both treatments (96.9% for AS/AQ and 100% for AL). In this study, the excellent efficacies observed with AS/AQ and AL at their present dosages seem to demonstrate good activity against the asexual forms of the parasite. The results of this study confirmed the policy decision of using AS/AQ and AL in Cameroon.

Parasitological cure rates have ranged from 94 to 100% in young African children. Studies conducted in Kenya Senegal and Gabon (three African countries with different patterns of malaria transmission and rates of chloroquine and amodiaquine resistance) reported high cure rates (>80%) for a 6-dose regimen of AL and a 3-day course of AS/AQ but fell short of therapeutic efficacy levels reported in other areas [18]. High therapeutic efficacies and the ranking (AL followed by AS/AQ) similar to those presently reported have previously been observed in (Uganda [19], Gabon [20], Southern Tanzania [21], Angola [22]), and many other African countries. Studies in Thailand have also shown that a six-dose regimen of AL is required in areas with multidrug-resistant *P. falciparum *to achieve an efficacy greater than 95% [23]. These data together now supports the wide deployment of these two artemisinin-based combinations in most endemic countries.

The article "Amodiaquine-Artesunate versus Artemether-Lumefantrine against Uncomplicated Malaria in Children Less Than 14 Years in Ngaoundere, North Cameroon: Efficacy, Safety, and Baseline Drug Resistant Mutations in pfcrt, pfmdr1, and pfdhfr Genes" was retracted in 2019. Reasons: errors in the methods; no approval from the institution; no approval from a third party.

### 4.2. Secondary Outcomes

The secondary outcomes of rapid fever-clearance, parasite-clearance, and the beneficial effect on blood haemoglobin levels were similar for the two therapies. This study has shown rapid parasite and fever clearance in children treated with 6-dose regimen of AL and 3-day course of AS/AQ. There was no clinical significant difference in efficacy between AL and the combination of AS/AQ. Similar patterns in parasite and fever clearance in Nigerian children have also been reported [24].

In terms of clinical parameters, both drugs were well tolerated by the patients. Drug-induced vomiting requiring retreatment was confined to a very small number of patients in both groups. Only minor adverse events were observed, as recorded in other studies with these same drugs [25, 26] and these did not require premature termination of treatment or specific medical care. All adverse events disappeared at the end of treatment and no serious adverse event was observed. This observation is most likely a reflection of the fact that most of the observed AEs were related to malaria symptoms, and the better efficacy associated with the study drugs allowed a more rapid resolution of malaria and thus prevented worsening of symptoms.

Despite the good parasitological efficacy in the two treatment groups, treatment did not produce complete haematological recovery. This may have been due to a combination of a relatively high mean, pretreatment haematocrit, the effect of artesunate on reticulocytes, and the relatively short follow-up period (28 days). Haematological recovery often requires more than four weeks in some malaria settings [27].

Biological tolerability was good for all drug combinations. Two serious complications of amodiaquine described in published studies are drug-induced hepatitis and neutropenia. Risk estimates, based on weekly amodiaquine prophylaxis, are 1 in 15,650 and 1 in 2000 for these two disorders, respectively [28]. No cases of clinical hepatitis were observed in the present study. However, it should be noted that our sample size was small and intended use was not prophylaxis but case active case management. There was a slight decline in neutrophil counts in some children from both study groups. A small number of participants developed neutropenia without clinical symptoms. Published data on amodiaquine-related neutropenia and hepatitis are few [29–31]. Cases with leukopenia (as a surrogate marker of neutropenia), anaemia, lymphopenia, and thrombocytopenia were also detected in the two treatment groups. Previous studies did not report changes in the total white cell or neutrophil counts [32, 33], while leukopenia and neutropenia have been previously described with AQ use [9]. In our study, the overall frequencies of leukopenia (17.6% versus 18.8%) and neutropenia (2.9% versus 13.0%) for the AS/AQ and AL treatment groups, respectively, were found to be higher than those reported by Schellenberg et al. [34] (leukopenia 3.7% and neutropenia 2.5% in AQ-treated Tanzanian children) and by Adjuik et al. (“unremarkable changes in WBC” but similar figures for severe neutropenia, namely, 6% in AQ or AQ plus AS treated African children) [18]. We cannot definitively ascribe the cause of neutropenia and leukopenia in our patients to amodiaquine because malaria itself could be a factor. Nevertheless, this finding calls for further studies to assess the safety and to define the risk-benefit ratio of repeated amodiaquine or AS/AQ use.

The article "Amodiaquine-Artesunate versus Artemether-Lumefantrine against Uncomplicated Malaria in Children Less Than 14 Years in Ngaoundere, North Cameroon: Efficacy, Safety, and Baseline Drug Resistant Mutations in pfcrt, pfmdr1, and pfdhfr Genes" was retracted in 2019. Reasons: errors in the methods; no approval from the institution; no approval from a third party.

This study also showed a lower proportion of patients with raised ALT >37 mg/dL than Schellenberg et al. 1.5 versus 3.0% [34]. The higher frequencies of laboratory-observed adverse events could be explained by comorbidities or pharmacogenetic differences in the study groups which we did not investigate in this study. Although there were no apparent clinical consequences of the haematological and biochemical changes in both study groups, the findings of the present study are a reminder that these AQ-related toxicities can occur after only one treatment. The consequences of its repeat use, especially in areas of intense transmission, needs careful monitoring following massive deployment [10]. Strategies for implementing an antimalarial pharmacovigilance program in Cameroon are therefore urgently needed. This is important because ACTs consumption is expected to increase since the therapy is now free to children less than five years old. It is also subsidised for all other age groups and distributed through many public drug outlets. This urgency is even more acute because of Cameroon's ongoing strategy of large scale deployment of ACTs for community management of RDT confirmed malaria by community health workers.

High levels of resistance conferring mutations to chloroquine and sulphadoxine-pyrimethamine circulate in the region of Ngaoundere. This confirms earlier findings about high *in vivo* CQ resistance and the decision whereby CQ is withdrawn from official use in treatment of malaria in Cameroon. Recent reports linking *pfmdr1* mutations and ACTs sensitivity [35] requires follow up because of the prevalence of *pfmdr1* mutations in this region. Future monitoring of molecular markers in distinct geographical regions of Cameroon are therefore warranted.

The article "Amodiaquine-Artesunate versus Artemether-Lumefantrine against Uncomplicated Malaria in Children Less Than 14 Years in Ngaoundere, North Cameroon: Efficacy, Safety, and Baseline Drug Resistant Mutations in pfcrt, pfmdr1, and pfdhfr Genes" was retracted in 2019. Reasons: errors in the methods; no approval from the institution; no approval from a third party.

## 5. Conclusion

According to the recommended malaria treatment policy, both AS/AQ and AL are suitable drugs for first-line purpose since both drugs recorded excellent PCR-corrected efficacies (i.e., 96.4% and 100%, resp.) and safety/tolerability profiles in children in this study. AL, however, appeared better than AS/AQ for several outcomes such as rapid parasitological clearance, resolution of symptoms, and biological tolerance. Pharmacovigilance research is needed to monitor safety following extensive deployment, especially when the use is indicated for pregnant women and for those with malaria comorbidities who constitute another vulnerable group.

## Figures and Tables

**Figure 1:** Kaplan Meier curve of the PCR adjusted efficacy outcome of treatment with either AS/AQ or AL during 28 days of followup. Assessment was per protocol and protocol violations were censored from the survival analysis.

**Figure 2:** Evolution of febrile patients following ingestion of AS/AQ and AL during 28 days of followup. During the trial period, fever, measured by adjusted axillary temperatures >37.5°C, was estimated daily during the first three days and subsequently during the trial protocol days and any other day the child felt unwell. There was no significant difference in fever clearance between trial groups (*P* > 0.05).

**Figure 3:** Evolution of parasite clearance in patients on treatment with AS/AQ or AL during 28 days of followup. Parasite clearance was measured daily for the first three days, and then on every other day including during regular appointments. Parasite load was estimated by microscopy in Giemsa stained thick blood smears. Within the first three days of ingestion of medication, parasite clearance was not different between treatments but was observed to be significantly lower in children on AS/AQ after day 7 (*P* < 0.001).

**Figure 4:** (a) and (b) show the prevalence of haplotypes of the dhfr and pfcrt genes in Ngaoundere, a savannah region in the north of Cameroon. IRN represents the fansidar resistance conferring mutant in the *dhfr* gene, NCS represent the wild type haplotype, and mixed haplotype is also represented. These haplotypes were built based on the presence of absence of mutation in codon 76 of the *pfcrt *gene (a) or cumulative mutations at codons 51, 59, and 108 of the *dhfr *gene (b).

The article "Amodiaquine-Artesunate versus Artemether-Lumefantrine against Uncomplicated Malaria in Children Less Than 14 Years in Ngaoundere, North Cameroon: Efficacy, Safety, and Baseline Drug Resistant Mutations in pfcrt, pfmdr1, and pfdhfr Genes" was retracted in 2019. Reasons: errors in the methods; no approval from the institution; no approval from a third party.

**Table 1:** Study participant's characteristics at enrolment.

Characteristic	AS/AQ (*n* = 73)	AL (*n* = 77)	*P* value
Sex			
Male	39 (53.4)	39 (50.6)	0.73
Female	34 (46.6)	38 (49.4)	
Age (years)			
Mean ± SD	04.93 ± 03.64	04.94 ± 03.32	0.98
Range	01.0–13.0	01.0–13.0	
Weight (kg)			
Mean ± SD	16.87 ± 08.36	16.06 ± 06.95	0.52
Range	07.0–41.0	06.0–35.0	
Temperature (°C)			
Mean ± SD	37.95 ± 01.19	37.91 ± 0.79	0.80
Range	31.1–40.5	35.5–39.8	
Haemoglobin (g/dL)			
Mean ± SD	10.63 ± 2.65	10.38 ± 2.42	0.55
Range	4.8–28.0	4.9–17.8	
Anaemia			
(Hb < 9.5 g/dL)	21/73 (28.8)	26/77 (33.8)	0.51
Parasitaemia (/*μ*L)			
GMPD	4628.30	3886.36	0.18
Range	1340–184 000	1240–156 000	

SD: standard deviation, GMPD: geometric mean parasite density, and numbers in brackets represent percentages. There were no significant differences between baseline characteristics for participants randomised in both treatment arms.

**Table 2:** Crude and PCR adjusted days 14 and 28 treatment outcomes of study participants on AS/AQ or AL.

Efficacy outcome	AS/AQ		AL	
	*N*	%	*N*	%
Crude day 14 cure rates	68		69	
ACPR	61	89.7	67	97.1
ETF	02	02.9	0	0
LCF	01	01.5	0	0
LPF	04	06.0	02	03.0
Crude day 28 cure rates	61		64	
ACPR	54	88.5	62	96.9
ETF	02	03.3	0	0
LCF	01	01.6	0	0
LPF	04	06.6	02	03.1
PCR corrected day 28 cure rates	56		62	
ACPR	54	96.4	62	100
ETF	02	03.6	0	0
LCF	0	0	0	0
LPF	0	0	0	0

Note: Reinfections were excluded from the analysis after profiling pretreatment and recurrent parasites based on the polymorphic *Plasmodium falciparum  msp  2* antigen. ACPR: adequate clinical parasitological response, ETF: early treatment failure, LCF: late clinical failure, LPF: late parasitological failure, and CI: confidence interval. Early treatment failures were noted in two patients randomized to receive ASAQ coblister. It was unclear if this was due to poor drug absorption or real treatment failures.

**Table 3:** Incidence of biological markers of adverse events in patients on AS/AQ or AL during 28 days of followup.

Laboratory parameter	AS/AQ		AL	
	*N*	%	*N*	%
Biochemistry				
Bilirubin > 1 mg/dL	20/68	29.4	18/69	26.1
Alanine transaminase > 37 mg/dL	01/68	01.5	0	0
Creatinine > 11 mg/dL	0		01/69	01.4
Haematology				
Anaemia (Hb < 9.5 g/dL)	23/68	33.8	21/69	30.4
Leucopenia (WBC < 5000/*μ*L)	12/68	17.6	13/69	18.8
Lymphopenia (lymph < 4.0)	10/68	14.7	10/69	14.5
Neutropenia (neutro < 1.5)	02/68	02.9	09/69	13.0
Platelets (platelets < 150∗10^3^)	02/68	02.9	03/69	04.3

**Table 4:** Mean variation in haematological and biochemical indices 14 days after treatment.

Parameter	AS/AQ			AL		
	*N*	Mean ± SD	Paired *t*-test	*N*	Mean ± SD	*P* value^+^
Haematocrit (%)						
D0	68	32.47 ± 04.92		69	33.59 ± 7.30	
D14	68	32.58 ± 05.31	0.87	69	33.24 ± 5.33	0.66
WBCs (×10^3^/*μ*L)						
D0	68	11.04 ± 06.72		69	12.78 ± 14.88	
D14	68	09.10 ± 05.38	0.04*	69	08.70 ± 4.13	0.026*
Platelets (×10^3^/*μ*L)						
D0	68	386.46 ± 326.96		69	466.50 ± 409.90	
D14	68	650.94 ± 508.88	0.001*	69	725.84 ± 609.51	0.002*
ALAT (U/L)						
D0	68	12.12 ± 11.23		69	12.86 ± 13.32	
D14	68	10.20 ± 08.03	0.25	69	10.52 ± 6.49	0.17
Creatinine (mg/L)						
D0	68	03.49 ± 2.07		69	3.68 ± 1.67	
D14	68	03.92 ± 2.01	0.17	69	4.51 ± 2.69	0.019*
Bilirubin (mg/L)						
D0	68	0.86 ± 0.80		69	0.99 ± 0.94	
D14	68	0.87 ± 0.86	0.95	69	0.86 ± 0.94	0.43

Indices were measured at pre-treatment and on day 14. Values are reported as mean readings ± standard deviation of patients treated with AS/AQ or AL.

The article "Amodiaquine-Artesunate versus Artemether-Lumefantrine against Uncomplicated Malaria in Children Less Than 14 Years in Ngaoundere, North Cameroon: Efficacy, Safety, and Baseline Drug Resistant Mutations in pfcrt, pfmdr1, and pfdhfr Genes" was retracted in 2019. Reasons: errors in the methods; no approval from the institution; no approval from a third party.

*N*: number, SD: standard deviation, ALAT: alanine transaminase, and *significant at threshold of *P* = 0.05. ^+^Paired students' *t*-test.
